# Post-Intake of *S*-Ethyl Cysteine and *S*-Methyl Cysteine Improved LPS-Induced Acute Lung Injury in Mice

This article has been retracted.

**DOI:** 10.3390/nu8080507

**Published:** 2016-08-19

**Authors:** Te-chun Hsia, Mei-chin Yin

**Affiliations:** 1 Department of Respiratory Therapy, China Medical University, Taichung City 40402, Taiwan; derrick.hsia@msa.hinet.net; 2 Department of Internal Medicine, China Medical University Hospital, Taichung City 40402, Taiwan; 3 Department of Nutrition, China Medical University, 91, Hsueh-shih Rd., Taichung City 40402, Taiwan; 4 Department of Health and Nutrition Biotechnology, Asia University, Taichung City 41354, Taiwan

**Keywords:** *S*-ethyl cysteine, *S*-methyl cysteine, lung, LPS, inflammation

## Abstract

The effects of *S*-ethyl cysteine (SEC) and *S*-methyl cysteine (SMC) on lipopolysaccharide (LPS)-induced acute lung injury in mice were examined. Eight hours after LPS challenge, SEC or SMC was supplied in drinking water at 0.5% or 1% for 3 days. LPS increased lung myeloperoxidase activity, neutrophil counts and edema. SEC or SMC post-intake attenuated these events. SEC or SMC suppressed LPS-induced lung expression of cyclooxygenase-2, nuclear factor-κB and mitogen-activated protein kinase, and lowered the generation of tumor necrosis factor-alpha, monocyte chemoattractant protein-1 and prostaglandin E_2_. LPS enhanced the expression of p47^phox^, gp91^phox^, Bax and cleaved caspase-3, and increased the production of reactive oxygen species in the lung. SEC or SMC post-intake reversed these alterations. These findings suggest that these agents could protect the lung through their anti-inflammatory, anti-oxidative and anti-apoptotic activities.

## 1. Introduction

Acute lung injury (ALI), a complicated respiratory disorder with a high morbidity rate, is characterized by pulmonary edema, inflammation, alveolar barrier disruption, capillary leak and hypoxemia [1,2]. It is reported that nuclear factor-κB (NF-κB) and mitogen-activated protein kinase (MAPK) signaling pathways play crucial roles in the inflammatory progression of ALI, and the activation of these pathways promotes the excessive release of cytokines and chemokines including interleukin (IL)-6, tumor necrosis factor (TNF)-alpha and monocyte chemoattractant protein (MCP)-1 [3,4]. In addition, the activation of cyclooxygenase (COX)-2 and the generation of prostaglandin E_2_ (PGE_2_) are also involved in the inflammatory deterioration and immune abnormality of ALI [5,6]. On the other hand, redox imbalance from NADPH oxidase activation is another important pathological feature of ALI, which causes reactive oxygen species (ROS) overproduction, depletes glutathione (GSH) and exacerbates lung oxidative injury [7]. The studies of Aggarwal et al. [8] and Wang et al. [9] revealed that ALI-associated lung cell death was highly related to the mitochondrial intrinsic apoptotic pathway, which was mainly regulated by the BLC family including anti-apoptotic and pro-apoptotic molecules. Obviously, the activation of these above pathways promotes apoptotic, oxidative and inflammatory stress in the lung, and finally leads to respiratory failure and even death. Thus, there is a need to develop agent(s) with anti-inflammatory, anti-apoptotic and anti-oxidative activities in order to increase therapeutic options for ALI.

An ALI animal model could be created by lipopolysaccharide (LPS) administration because LPS caused abnormal immune response, stimulated the formation of ROS and inflammatory mediators such as TNF-alpha and PGE_2_ in lung and airway epithelial cells [10]. Yeh et al. [11] indicated that LPS decreased lung activity of glutathione peroxidase (GPX), catalase and heme oxygenase-1, which in turn diminished the anti-oxidative defensive capability of the lung. So far, the LPS-induced ALI model has been widely used for studies associated with lung protection or therapy [12].

*S*-ethyl cysteine (SEC) and *S*-methyl cysteine (SMC) are hydrophilic cysteine-containing compounds naturally synthesized in many *Allium* plant foods such as garlic and onion [13]. It has been reported that garlic extract protected lung and bronchial smooth muscle cell lines via increasing intracellular GSH content [14]. Our previous animal study found that dietary intake of SEC or SMC displayed anti-oxidative and anti-inflammatory protection against ethanol-induced liver injury in mice [15]. Our other study indicated that SEC or SMC ameliorated H_2_O_2_-induced apoptotic, oxidative and inflammatory injury in human BEAS-2B cells (bronchial cells) through preserving Bcl-2 expression, decreasing ROS formation and limiting protein expression of NAPDH oxidase, NF-κB and MAPK [16]. Those previous studies suggest that SEC and SMC are agents with anti-oxidative and anti-inflammatory activities, and may be able to protect the lung. Thus, an animal study was then conducted to investigate the therapeutic effects of SEC or SMC in the lung against LPS-induced injury.

In our present study, LPS was used to induce ALI. The effects of SEC or SMC post-treatments at various doses upon pulmonary edema, neutrophils counts and myeloperoxidase (MPO) activity were examined. The impact of these agents upon protein expression of COX-2, NF-κB, MAPK, NADPH oxidase and Bcl-2 in the lung was evaluated.

## 2. Materials and Methods

### 2.1. Materials

SEC and SMC (99%) were purchased from Wako Chemical Co. (Tokyo, Japan). LPS (*Escherichia coli* 055:B5) was obtained from Sigma-Aldrich Co. (St. Louis, MO, USA).

### 2.2. Animals

Male Balb/cA mice, 3–4 week old, were purchased from the National Laboratory Animal Center (Taipei City, Taiwan). Mice were housed on a schedule of 12-h light/dark. The use of mice was reviewed and approved by the China Medical University animal care committee, and the permission number was 2016-033. Mice with body weight at 25.4 ± 1.2 g were used.

### 2.3. Experimental Design

SEC or SMC at 0.5 g or 1 g was mixed with 99.5 or 99 mL distilled water to prepare low or high dose groups. Mice were divided into six groups: normal group, LPS group, LPS + low SEC group, LPS + high SEC group, LPS + low SMC group and LPS + high SMC group. Each group had ten mice. Mice were anesthetized by diethyl ether inhalation, and followed by intranasally injecting LPS, 10 μg in 50 μL phosphate buffer saline (PBS), to induce ALI. Eight hours after LPS administration, SEC or SMC was supplied in drinking water. All mice had free access to food and water at all times. Body weight, consumed feed and water were recorded. After 3 days of supplement, mice were sacrificed with carbon dioxide. Blood and lungs were collected. Plasma was immediately separated from erythrocyte. The activity of alanine aminotransferase (ALT) and aspartate aminotransferase (AST) in plasma was measured by kits purchased from Randox Laboratories Ltd. (Crumlin, UK). Bronchoalveolar lavage fluid (BALF) was collected by washing the airways of right lungs three times with PBS through a tracheal cannula, 0.5 mL PBS each time. After centrifugation at 500× *g*, 10 min at 4 °C, supernatant was used for neutrophil counts. Lung at 50 mg was homogenized in cold PBS and the filtrate was collected. The protein concentration of lung filtrate was determined by an assay kit (Pierce Biotechnology Inc., Rockford, IL, USA), and bovine serum albumin was used as a standard.

### 2.4. Lung Wet/Dry Weight Ratio

The fresh middle lobe of the right lungs was weighed, which was defined as wet weight. Lung tissue was then placed in an oven for 48 h at 80 °C, and the weight was defined as dry weight. The ratio of lung wet/dry (W/D) weight was calculated to evaluate pulmonary edema.

### 2.5. MPO Activity Assay

MPO activity reflects the infiltration of neutrophils into the lung, and was measured according to the method of Choi et al. [17]. Briefly, lung tissue was homogenized and centrifuged. Pellet was re-suspended in 50 mM PBS containing 0.5% hexadecyltrimethylammonium bromide. After centrifugation, the pellet was re-suspended and reacted with 3,3′,5,5′-tetramethylbenzidine, and followed by incubating at 37 °C for 2 min. Reaction was terminated by adding 100 μL 2 mM H_2_SO_4_. The absorbance at 450 nm was recorded. MPO activity was shown as unit/per mg protein.

### 2.6. Determination of Inflammatory Factors

Lung tissue was homogenized in 10 mM Tris-HCl buffered solution (pH 7.4) containing 2 M NaCl, 1 mM EDTA, 0.01% Tween 80, 1 mM phenylmethylsulfonyl fluoride. After centrifugation at 9000× *g* at 4 °C for 30 min, the supernatant was collected and used for cytokine measurement. The levels of IL-1beta, IL-6, TNF-alpha and MCP-1 were determined by ELISA using cytoscreen immunoassay kits (BioSource International, Camarillo, CA, USA). The detection limit was 10 pg/mg protein for TNF-alpha and MCP-1, and 5 pg/mg protein for IL-1beta and IL-6. PGE_2_ level was determined by a PGE_2_ EIA kit obtained from Cayman Chemical Co. (Ann Arbor, MI, USA).

### 2.7. Measurement of Oxidative Factors

GSH or oxidized glutathione (GSSG) concentration (nmol/mg protein) in lung homogenate was quantified by colorimetric GSH or GSSG assay kit (OxisResearch, Portland, OR, USA). The activity (U/mg protein) of GPX, glutathione reductase (GR) or catalase was assayed by commercial kit (Calbiochem Inc., San Diego, CA, USA). ROS level was measured according to the method of Ali et al. [18]. Lung tissue was homogenized on cold PBS buffer containing EDTA. An oxidation sensitive dye, 2′,7′-dichlorofluorescein diacetate, at 25 mM was added to homogenates. After 30 min incubation, fluorescence change was measured by a fluorescence microplate reader with excitation wavelength at 480 nm and emission wavelength at 535 nm.

### 2.8. Western Blot Analyses

Partial lung tissue was homogenized in buffer containing protease-inhibitor cocktail (1:1000) and 0.5% Triton X-100. After determining protein content, each sample at 40 μg protein was used for SDS-polyacrylamide gel electrophoresis, and transferred to a nitrocellulose membrane for 1 h. A solution containing nonfat milk was added, and followed by incubating for another 1 h to prevent non-specific binding of antibody. Membrane was then reacted with monoclonal antibody against Bcl-2, Bax, cleaved caspase-3, p47^phox^, gp91^phox^, GPX, GR and catalase (1:2000), COX-2, NF-κB p50, NF-κB p65 or MAPK (1:1000) at 4 °C overnight, and further treated with horseradish peroxidase conjugated antibody for 3.5 h at 25 °C. The detected bands were processed by an image analyzer, and the blot was quantified and normalized against glyceraldehyde-3-phosphate dehydrogenase (GAPDH), which was used for loading control.

### 2.9. Statistical Analyses

Data were expressed as mean ± standard deviation (SD), and *n* = 10. Statistical analyses were processed by one-way analysis of variance. Furthermore, Dunnett’s *t*-test was used for post-hoc comparison. Statistical significance is defined as *p* < 0.05.

## 3. Results

### 3.1. Effects of SEC and SMC on MPO and Neutrophil Counts

LPS administration decreased body weight and increased lung W/D ratio (Table 1, *p* < 0.05). SEC or SMC post-intake at 0.5% or 1% reversed these changes (*p* < 0.05). LPS, SEC or SMC treatments did not affect plasma ALT and AST activities (*p* > 0.05). As shown in Figure 1, LPS increased lung MPO activity and BALF neutrophil counts (*p* < 0.05). SEC or SMC post-intake at both doses lowered MPO activity and neutrophil counts (*p* < 0.05), in which SMC at 1% exhibited the greatest effects in reducing MPO activity and neutrophil counts (*p* < 0.05). SMC at 0.5% displayed similar effects as 1% SEC in decreasing MPO activity and neutrophil counts (*p* > 0.05).

### 3.2. Effects of SEC and SMC on Inflammatory Factors

LPS stimulated the production of IL-1beta, IL-6, TNF-alpha, MCP-1 and PGE_2_ (Table 2, *p* < 0.05). SEC or SMC post-intake at both doses decreased the release of these inflammatory factors, in which SMC at 1% was greater than SEC at the same dose in lowering lung IL-1beta, IL-6 and MCP-1 levels (*p* < 0.05). LPS up-regulated the expression of COX-2, NF-κB and MAPK in lung (Figure 2, *p* < 0.05). SEC and SMC at both doses suppressed lung expression of COX-2, NF-κB p50, NF-κB p65 and p-p38 (*p* < 0.05). SMC post-intake at 1% led to less COX-2 and p-p38 expression than SEC at equal dose (*p* < 0.05).

### 3.3. Effects of SEC and SMC upon Oxidative and Apoptotic Factors

As shown in Table 3, LPS depleted GSH content, increased GSSG and ROS levels, and decreased the activity of GPX, GR and catalase in the lung (*p* < 0.05). SEC or SMC post-intake at both doses reversed these alterations (*p* < 0.05). SEC at 1% led to higher GSH content and lower ROS level than SMC at 1% (*p* < 0.05). LPS enhanced lung expression of p47^phox^ and gp91^phox^, and suppressed lung expression of GPX, GR and catalase (Figure 3, *p* < 0.05). SEC or SMC post-intake at both doses down-regulated the expression of p47^phox^ and gp91^phox^, in which SEC at 1% led to less p47^phox^ and gp91^phox^ expression than SMC at 1% (*p* < 0.05). SEC or SMC post-intake promoted lung expression of GPX, GR and catalase (*p* < 0.05), and dose-dependent manner was presented in up-regulating GR expression (*p* < 0.05). LPS suppressed Bcl-2 expression, and increased the expression of Bax and cleaved caspase-3 in lung (Figure 4, *p* < 0.05). SEC or SMC post-intake decreased lung Bax and cleaved caspase-3 expression, and dose-dependent effect was shown in lowering Bax expression (*p* < 0.05). SEC or SMC post-intake also raised lung Bcl-2/Bax ratio (*p* < 0.05).

## 4. Discussion

Our previous cell line study revealed that pre-treatments of SEC or SMC, two cysteine-containing compounds, protected human bronchial cells against H_2_O_2_-induced damage [16]. The results from our present animal study further found that post-intake of SEC or SMC markedly improved LPS-induced inflammatory, oxidative and apoptotic lung injury through decreasing MPO activity and neutrophil counts, and declining NF-κB, MAPK and NADPH oxidase pathways. A schematic diagram for lung protein from these two agents against LPS is shown in Figure 5. These findings support the notion that SEC and SMC improve the defensive capability of respiratory system.

Pulmonary edema, an important pathological feature of ALI, could be evaluated by lung W/D weight ratio in animal ALI model [19]. In our present study, SEC or SMC post-intake effectively attenuated pulmonary edema in those mice, which was evidenced by lower W/D weight ratios. Neutrophils could be activated by inflammatory insult, like LPS, and migrate to the site of injury, where they undergo defensive actions via degranulation, phagocytosis and ROS generation [20]. Furthermore, activated neutrophils act as signaling indicators to promote inflammatory response and enhance the production of additional cytokines in local and/or systemic levels [21]. MPO is involved in the microbicidal activity of neutrophils [22], and its activity reflects the activation and recruitment of neutrophils into lung [23]. As reported by others [24] and our present study, LPS caused ALI-like immune abnormality, which was evidenced by increased MPO activity and neutrophil counts. However, we found that SEC or SMC post-intake markedly lowered BALF neutrophil counts and lung MPO activity in LPS-treated mice. The less neutrophil counts suggest that lung-immune hyper-responsiveness due to LPS stimulation has been reduced by these two agents, which in turn alleviates inflammatory response and leads to lower cytokines and ROS formation. MCP-1 is a chemokine responsible for recruiting monocytes and other inflammatory cells to the sites of tissue injury [25]. It is reported that monocyte activation participated in LPS-induced ALI progression [26]. Our data agreed that monocyte infiltration was involved in LPS-induced ALI because of the higher MCP-1 levels. However, we observed that SEC or SMC post-intake decreased lung MCP-1 content, which implied that these compounds ameliorated ALI via diminishing monocytes infiltration. The reduction of neutrophil and monocyte activation by SEC or SMC indicated that these compounds attenuated LPS-induced abnormal immune functions in the lung.

It is well known that LPS activated lung NF-κB and MAPK pathways, which consequently raised lung inflammatory stress by stimulating excessive production of IL-1beta, IL-6 and TNF-alpha [3,11]. We found SEC or SMC post-intake down-regulated LPS-induced lung expression of NF-κB p50 and NF-κB p65, as well as limited p38 phosphorylation, which led to a decrease in the generation of these inflammatory cytokines. This evidence indicated that these two compounds improved LPS-caused lung inflammation via suppressing NF-κB and MAPK pathways. In addition, COX-2 is highly expressed in lung under some pathological conditions like ALI, and it is responsible for the production of lipid inflammatory mediator such as PGE_2_ [27]. PGE_2_ is a potent bronchodilator and also a regulator for macrophage activation [28]. Thus, agent with the effect to inhibit COX-2 protein expression and PGE_2_ formation could be considered a potent therapeutic choice for inflammatory diseases [29]. In our present study, SEC or SMC post-intake effectively down-regulated LPS-induced COX-2 expression, which consequently reduced PGE_2_ biosynthesis. Apparently, the anti-inflammatory protection from SEC or SMC against LPS-induced ALI was partially due to the inhibition of these compounds upon COX-2/PGE_2_ pathway.

NADPH oxidase complex plays a key role for ROS formation in respiratory disorders including ALI [30]. gp91^phox^ and p47^phox^ are membrane and cytosolic component of NADPH oxidase, respectively. SEC and SMC post-intake substantially restricted lung protein expression of gp91^phox^ and p47^phox^, which subsequently decreased ROS production and mitigated lung oxidative stress. Apparently, SEC or SMC could improve LPS-induced oxidative lung injury via suppressing the NADPH oxidase pathway. In addition, SEC or SMC post-intake also increased both activity and protein expression of GPX, GR and catalase in the lungs of LPS-treated mice, which definitely contributed to enhanced anti-oxidative lung defense and alleviated LPS-induced oxidative injury. Moreover, the increased activity and expression of GPX and GR from SEC or SMC treatments improved the conversion of GSSG to GSH. Thus, greater GSH content and lower GSSG levels in the lungs of SEC or SMC treated mice could be explained. These results revealed that the anti-oxidative protection from SEC or SMC could be partially ascribed to these compounds maintaining glutathione homeostasis. LPS promoted the lung’s mitochondrial intrinsic apoptotic pathway, which was evidenced by lower Bcl-2 expression and greater Bax and cleaved caspase-3 expression, as we observed. Although SEC or SMC post-intake failed to up-regulate the expression of Bcl-2, an anti-apoptotic molecule, both compounds substantially limited the expression of Bax and cleaved caspase-3, two crucial pro-apoptotic molecules, which consequently ameliorated lung apoptotic injury. The increased ratio of Bcl-2/Bax also suggested that both compounds attenuated LPS-induced lung apoptotic stress.

It is interesting to find that SEC exhibited greater effects in increasing GSH content and decreasing ROS level, but SMC was greater in lowering neutrophils, MPO activity, cytokines levels and protein expression of COX-2 and p-p38. It is highly possible that the action modes of these two compounds are not identical although their structures are similar. SEC and SMC are naturally synthesized in *Allium* plants such as onion and garlic. The doses used in mice, 0.5% or 1%, are approximately equal to 28 or 56 grams for adults with 70-kg body weight. Our data regarding plasma ALT and AST activities supported the notion that these two agents at these doses did not impair hepatic functions. Based on their natural and edible properties, the application of SEC or SMC for ALI therapy may be feasible and safe.

In conclusion, *S*-ethyl cysteine and *S*-methyl cysteine post-intake for 3 days improved LPS-induced, acute inflammatory, oxidative and apoptotic injury in the lung through inactivating neutrophils and monocytes, and limiting protein expression of COX-2, NF-κB, p-p38, NADPH oxidase and Bax. These findings suggest that these agents could aid ALI therapy.

## Figures and Tables

**Figure 1:** Lung MPO (myeloperoxidase) activity (**a**); and neutrophil count (**b**) of mice in normal group, LPS (lipopolysaccharide) group, LPS + low SEC (*S*-ethyl cysteine) group, LPS + high SEC group, LPS + low SMC (*S*-methyl cysteine) group and LPS + high SMC group after 3-day treatments. Data are mean ± SD (standard deviation), *n* = 10. ^a–e^ Means among bars without a common letter differ, *p* < 0.05.

**Figure 2:** Lung expression of COX-2, NF-κB and MAPK of mice in normal group, LPS group, LPS + low SEC group, LPS + high SEC group, LPS + low SMC group and LPS + high SMC group after 3-day treatments. Data are mean ± SD, *n* = 10; ^a−e^ Means among bars without a common letter differ, *p* < 0.05.

**Figure 3:** Lung expression of p47^phox^, gp91^phox^, GPX, GR and catalase of mice in normal group, LPS group, LPS + low SEC group, LPS + high SEC group, LPS + low SMC group and LPS + high SMC group after 3-day treatments. Data are mean ± SD, *n* = 10; ^a−e^ Means among bars without a common letter differ, *p* < 0.05.

**Figure 4:** Lung expression of Bcl-2, Bax and cleaved caspase-3, and ratio of Bcl-2/Bax of mice in normal group, LPS group, LPS + low SEC group, LPS + high SEC group, LPS + low SMC group and LPS + high SMC group after 3-day treatments. Data are mean ± SD, *n* = 10; ^a−d^ Means among bars without a common letter differ, *p* < 0.05.

**Figure 5:** Schematic diagram for lung protein of SEC or SMC against LPS.

**Table 1:** Water intake (WI, mL/mouse/day), feed intake (FI, g/mouse/day), body weight (BW, g/mouse), lung W/D (wet/dry) ratio, plasma ALT (activity of alanine aminotransferase) or AST (aspartate aminotransferase) activity (U/mg protein) of mice in normal group, LPS (lipopolysaccharide) group, LPS + low SEC (*S*-ethyl cysteine) group, LPS + high SEC group, LPS + low SMC (*S*-methyl cysteine) group and LPS + high SMC group after 3-day treatments. Data are mean ± SD (standard deviation), *n* = 10. ^a–d^ Means in a row without a common letter differ, *p* < 0.05.

	Normal	LPS	LPS + SEC, Low	LPS + SEC, High	LPS + SMC, Low	LPS + SMC, High
WI	2.3 ± 0.8 ^a^	1.9 ± 0.4 ^a^	2.1 ± 0.5 ^a^	2.0 ± 0.7 ^a^	1.8 ± 0.6 ^a^	2.1 ± 0.7 ^a^
FI	2.2 ± 0.5 ^a^	1.8 ± 0.6 ^a^	2.0 ± 0.4 ^a^	1.9 ± 0.6 ^a^	1.8 ± 0.4 ^a^	2.0 ± 0.5 ^a^
BW	26.1 ± 1.0 ^b^	22.9 ± 0.4 ^a^	24.9 ± 0.6 ^b^	25.5 ± 0.5 ^b^	24.7 ± 0.3 ^b^	25.3 ± 0.8 ^b^
W/D	2.8 ± 0.2 ^a^	6.4 ± 0.4 ^d^	5.3 ± 0.2 ^c^	3.9 ± 0.3 ^b^	5.0 ± 0.2 ^c^	3.7 ± 0.4 ^b^
ALT	27 ± 2 ^a^	35 ± 5 ^a^	32 ± 3 ^a^	28 ± 4 ^a^	29 ± 3 ^a^	25 ± 4 ^a^
AST	24 ± 4 ^a^	31 ± 2 ^a^	30 ± 4 ^a^	26 ± 5 ^a^	32 ± 4 ^a^	27 ± 3 ^a^

**Table 2:** Lung level of IL-1beta (interleukin) (pg/mg protein), IL-6 (pg/mg protein), TNF-alpha (tumor necrosis factor) (pg/mg protein), MCP-1 (pg/mg protein) (monocyte chemoattractant protein) and PGE_2_ (prostaglandin E_2_) (pg/g protein) of mice in normal group, LPS group, LPS + low SEC group, LPS + high SEC group, LPS + low SMC group and LPS + high SMC group after 3-day treatments. Data are mean ± SD, *n* = 10.

	Normal	LPS	LPS + SEC, Low	LPS + SEC, High	LPS + SMC, Low	LPS + SMC, High
IL-1beta	12 ± 3 ^a^	195 ± 14 ^e^	149 ± 9 ^d^	92 ± 11 ^c^	138 ± 13 ^d^	68 ± 6 ^b^
IL-6	10 ± 2 ^a^	218 ± 10 ^e^	161 ± 12 ^d^	101 ± 7 ^c^	153 ± 9 ^d^	57 ± 5 ^b^
TNF-alpha	13 ± 4 ^a^	253 ± 16 ^d^	192 ± 8 ^c^	112 ± 13 ^b^	188 ± 14 ^c^	97 ± 10 ^b^
MCP-1	15 ± 3 ^a^	231 ± 12 ^e^	174 ± 15 ^d^	116 ± 9 ^c^	165 ± 11 ^d^	82 ± 5 ^b^
PGE_2_	558 ± 49 ^a^	2271 ± 124 ^d^	1645 ± 110 ^c^	1082 ± 96 ^b^	1431 ± 108 ^c^	952 ± 73 ^b^

^a−e^ Means in a row without a common letter differ, *p* < 0.05.

**Table 3:** Lung level of GSH (nmol/mg protein), GSSG (nmol/mg protein), ROS (RFU/mg protein), and activity (U/mg protein) of GPX, GR and catalase of mice in normal group, LPS group, LPS + low SEC group, LPS + high SEC group, LPS + low SMC group and LPS + high SMC group after 3-day treatments. Data are mean ± SD, *n* = 10.

	Normal	LPS	LPS + SEC, Low	LPS + SEC, High	LPS + SMC, Low	LPS + SMC, High
GSH	19.1 ± 0.5 ^e^	8.1 ± 0.2 ^a^	11.3 ± 0.4 ^b^	16.0 ± 0.7 ^d^	11.1 ± 0.4 ^b^	13.9 ± 0.3 ^c^
GSSG	0.27 ± 0.05 ^a^	1.50 ± 0.16 ^d^	0.98 ± 0.09 ^c^	0.59 ± 0.06 ^b^	1.03 ± 0.08 ^c^	0.67 ± 0.07 ^b^
ROS	0.19 ± 0.04 ^a^	1.71 ± 0.14 ^e^	1.19 ± 0.11 ^d^	0.58 ± 0.09 ^b^	1.25 ± 0.12 ^d^	0.92 ± 0.1 ^c^
GPX	29.4 ± 2.3 ^d^	16.3 ± 1.4 ^a^	19.0 ± 1.2 ^b^	23.3 ± 1.6 ^c^	20.1 ± 0.8 ^b^	24.5 ± 1.3 ^c^
GR	1.82 ± 0.12 ^d^	0.67 ± 0.06 ^a^	1.02 ± 0.1 ^b^	1.38 ± 0.08 ^c^	0.95 ± 0.07 ^b^	1.31 ± 0.11 ^c^
catalase	22.8 ± 1.5 ^d^	12.7 ± 0.6 ^a^	15.9 ± 1.4 ^b^	19.0 ± 0.7 ^c^	15.1 ± 1.0 ^b^	18.6 ± 1.3 ^c^

^a−e^ Means in a row without a common letter differ, *p* < 0.05.
